The article "Intra-cardiac transfer of fatty acids from capillary to cardiomyocyte" was published in 2022. Journal: PLoS One.

# Intra-cardiac transfer of fatty acids from capillary to cardiomyocyte

**DOI:** 10.1371/journal.pone.0261288

**Published:** 2022-01-28

**Authors:** Ger J. van der Vusse, Theo Arts, James B. Bassingthwaighte, Robert S. Reneman

**Affiliations:** 1 Department of Physiology, Cardiovascular Research Institute Maastricht, Maastricht University, Maastricht, the Netherlands; 2 Center for Bioengineering, University of Washington, Seattle, Washington, United States of America; 3 Department of Biomedical Engineering, Cardiovascular Research Institute Maastricht, Maastricht University, Maastricht, the Netherlands; University of Jyvaskyla, FINLAND

## Abstract

Blood-borne fatty acids (*Fa*) are important substrates for energy conversion in the mammalian heart. After release from plasma albumin, *Fa* traverse the endothelium and the interstitial compartment to cross the sarcolemma prior to oxidation in the cardiomyocytal mitochondria. The aims of the present study were to elucidate the site with lowest *Fa* permeability (*i*.*e*., highest *Fa* resistance) in the overall *Fa* trajectory from capillary to cardiomyocyte and the relative contribution of unbound *Fa* (detach pathway, characterized by the dissociation time constant *τ*_*AlbFa*_) and albumin-bound *Fa* (contact pathway, characterized by the membrane reaction rate parameter *d*_*Alb*_) in delivering *Fa* to the cellular membranes. In this study, an extensive set of 34 multiple indicator dilution experiments with radiolabeled albumin and palmitate on isolated rabbit hearts was analysed by means of a previously developed mathematical model of *Fa* transfer dynamics. In these experiments, the ratio of the concentration of palmitate to albumin was set at 0.91. The analysis shows that total cardiac *Fa* permeability, *P*_*tot*_, is indeed related to the albumin concentration in the extracellular compartment as predicted by the mathematical model. The analysis also reveals that the lowest permeability may reside in the boundary zones containing albumin in the microvascular and interstitial compartment. However, the permeability of the endothelial cytoplasm, *P*_*ec*,_ may influence overall *Fa* permeability, *P*_*tot*_, as well. The model analysis predicts that the most likely value of *τ*_*AlbFa*_ ranges from about 200 to 400 ms. In case *τ*_*AlbFa*_ is fast, *i*.*e*., about 200 ms, the extracellular contact pathway appears to be of minor importance in delivering *Fa* to the cell membrane. If *Fa* dissociation from albumin is slower, *e*.*g*. *τ*_*AlbFa*_ equals 400 ms, the contribution of the contact pathway may vary from minimal (*d*_*Alb*_≤5 nm) to substantial (*d*_*Alb*_ about 100 nm). In the latter case, the permeability of the endothelial cytoplasm varies from infinite (no hindrance) to low (substantial hindrance) to keep the overall *Fa* flux at a fixed level. Definitive estimation of the impact of endothelial permeability on *P*_*tot*_ and the precise contribution of the contact pathway to overall transfer of *Fa* in boundary zones containing albumin requires adequate physicochemical experimentation to delineate the true value of, among others, *τ*_*AlbFa*_, under physiologically relevant circumstances. Our analysis also implies that concentration differences of unbound *Fa* are the driving force of intra-cardiac *Fa* transfer; an active, energy requiring transport mechanism is not necessarily involved. Membrane-associated proteins may facilitate *Fa* transfer in the boundary zones containing albumin by modulating the membrane reaction rate parameter, *d*_*Alb*_, and, hence, the contribution of the contact pathway to intra-cardiac *Fa* transfer.

## Introduction

To fulfil the energy requirements for electro-mechanical activity, the heart relies heavily on the uptake of blood-borne substrates. Although the heart can be considered to be an “omnivore”, under physiological conditions fatty acids (*Fa*) are the substrates of preference for cardiac energy conversion [1, 2]. Due to their very low solubility in water, *Fa* delivered to the heart are predominantly bound to plasma albumin [3]. Since the myocardial endothelium is virtually impermeable to albumin, *Fa* pass the microvascular endothelium after dissociation of the *Fa*-albumin complex followed by transfer to cardiomyocytes and metabolic conversion of *Fa* inside them [2]. In the endothelial cytoplasm, low-molecular weight Fatty Acid-Binding Proteins (*FABP*_*ec*_) are supposed to facilitate the intra-endothelial transfer of *Fa*. Subsequently, *Fa* diffuse through the peri-capillary interstitium predominantly bound to interstitial albumin, pass the cell membrane of the cardiomyocytes and diffuse through the cardiac muscle cytoplasm, facilitated by a muscle cell-specific *FABP*_*myo*_ [4].

Theoretically, in all fluid compartments two zones can be identified: a bulk zone far away from cell membranes, and a boundary zone, being the fluid layer in close vicinity to the cell membrane. A notable drop in the concentration of non-protein bound *Fa* characterizes this boundary zone [5]. *Fa* are delivered to cell membranes either by direct translocation of *Fa* from the *Fa*-binding protein (albumin or *FABP*), *i*.*e*., the so-called contact pathway, or preceded by release from the *Fa*-binding protein as free *Fa* in the aqueous solution, followed by free *Fa* diffusion towards and dissolution in the cell membrane, *i*.*e*., the so-called detach pathway [5]. Albumin serves as *Fa*-carrier protein in the extracellular boundary zones. The contribution of the detach pathway to overall intra-cardiac *Fa* transfer is determined by the dissociation time constant of the *Alb-Fa* complex, *τ*_*AlbFa*_, while the contribution of the detach pathway is governed by the membrane reaction rate parameter *d*_*Alb*_ (Fig 1).

**Fig 1:** Graph showing diffusion of free *Fa* and *Fa* bound to albumin through the fluid of the extra-cellular boundary zone in the capillary or interstitium towards a cell membrane, consisting of a phospholipid bilayer. In case *Fa* directly translocate from the *Alb*.*Fa* complex to the phospholipid bilayer, *i*.*e*, without first being released from the complex into the aqueous solution, the contact pathway is involved. Transfer of free *Fa* to the cell membrane occurs via the detach pathway in case *Fa* are released from the complex prior to diffusion through the aqueous solution and dissolution of the *Fa* moieties in the phospholipid bilayer. Unbound, *i*.*e*., *Fa* free, *Alb* diffuses back into the aqueous compartment. Note that all processes shown are reversible. *τ*_*AlbFa*_ and *d*_*Alb*_ refer to the dissociation time constant of the *AlbFa* complex and the membrane reaction rate parameter of the interaction of the *AlbFa* complex with the membrane, respectively.

Until now, it is incompletely understood which of the extra- or intracellular compartments has the highest resistance in the overall transfer pathway of *Fa* from capillary to the cardiomyocyte. Previously, the endothelial cells lining the microvascular compartment were proposed as the site of highest constraint [6]. However, it cannot be excluded that other fluid compartments such as the boundary zones in the capillary and in the peri-capillary interstitium, and the cardiac muscle cytoplasm may limit overall *Fa* transfer in the heart as well.

To gain better insight into the myocardial transfer of *Fa* previously we developed a mathematical model based upon standard physical and physicochemical principles, including diffusion-facilitating *Fa* carriers in the extra- and intracellular compartments [5]. The model allowed for experimental testing. The outcome of the test indicated that the model simulations compared favorably with data obtained in a small set of multiple indicator dilution experiments on isolated rabbit hearts [5]. In these comparisons, we were dealing with uncertainties regarding the values of parameters relevant for the albumin-related contact and detach pathways, represented by the membrane reaction rate parameter, *d*_*Alb*_, and the dissociation time constant of the albumin-fatty acid complex, *τ*_*AlbFa*_, respectively. Uncertainty also exists in the mathematical model about the *Fa*-permeability of the endothelial cytoplasm, *P*_*ec*,_. In the present study, we tried to shed more light on the values of the parameters *d*_*Alb*_, *τ*_*AlbFa*_, and *P*_*ec*_, using an extensive set of data obtained in 34 multiple indicator dilution experiments performed on isolated rabbit hearts. In these experiments, the hearts were perfused with a crystalline solution containing radiolabeled albumin and palmitate in varying concentrations, keeping the ratio between albumin and palmitate constant.

In analyzing the experimental data, we focused on the dependency of total permeability from capillary through endothelium and interstitium to the cardiomyocyte, *P*_*tot*_, on the total albumin concentration in the perfusate, [*Alb*], since the mathematical model indicated that there is a relationship between *P*_*tot*_ and [*Alb*] [5]. It is of note that *P*_*tot*_ is the resultant of the permeabilities of all boundary zones, cellular membranes and aqueous compartments, such as the endothelial and cardiac muscle cytoplasm, and the interstitium, to be crossed by *Fa* on their way from capillary to cardiomyocyte being the site of metabolic conversion.

By fitting the experimental findings with simulated data acquired with the mathematical model, we aimed at obtaining insight into: 1) the quantitative relationship between *P*_*tot*_ and the extra-cellular albumin concentration [*Alb*], 2) the range of physiologically and statistically acceptable values of the membrane reaction rate parameter, *d*_*Alb*_, the dissociation time constant of the albumin-fatty acid complex, *τ*_*AlbFa*_, and the endothelial *Fa*-permeability, *P*_*ec*_, 3) the relative impact of endothelial permeability, *P*_*ec*_, and the permeability of the albumin-containing boundary zone, *P*_*b*_, on overall *Fa*-permeability, *P*_*tot*_, and 4) the contribution of the contact pathway, relative to the detach pathway, to *Fa*-transfer in these boundary zones.

## Materials and methods

### Animal preparation

The study was performed in accordance with Guide for Care and use of laboratory animals published by the US National Institute of Health (NIH publication # 85–23). New Zealand adult male white rabbits (n = 9; 3.3 ± 0.4 kg body mass) were used. After induction of anesthesia with 40 mg sodium pentobarbital per kg body mass, injected into an ear vein in combination with heparin (500 U), the chest was opened by sternal thoracotomy. The heart was extirpated and rinsed in ice-cold Krebs-Ringer bicarbonate buffer to remove adherent blood. Total heart mass varied from 7.0 to 12.7 gram wet weight.

### Heart perfusion

The experiments were performed on isolated, non-ejecting, spontaneously beating hearts. To this end, the aortic stump of the hearts was mounted on the aortic inflow cannula of a custom-made Langendorff-perfusion apparatus. Perfusion via the aortic stump was started with oxygenated Krebs-Ringer-bicarbonate solution (KRB-buffer) for 10 min. Temperature of the heart was maintained at 36.5°C. Diastolic perfusion pressure was set at 50 mmHg. Heart rate ranged from 70 to 115 beats per min, but remained stable during each experiment. Perfusion pressure and heart rate were recorded continuously by means of a pressure transducer connected to the aortic inflow cannula and an ECG-recorder, respectively. A small catheter was inserted through the apex of the right ventricle to collect perfusate samples of fluid originating from the coronary sinus (see below). The left ventricle was drained routinely via a small cannula pierced through the apex to prevent loading of the left ventricle cavity by fluid from the Thebesian veins. Flow rates through both the right and left ventricular cannula were monitored with the use of a calibrated cylinder, prior to each tracer injection. Flow of the solution through the coronary bed of the left ventricle varied from 1.8 to 3.9 ml g^-1^ wet weight min^-1^ between experiments, but remained stable during any individual experiment.

Each heart (n = 9) was subsequently perfused with four different solutions, varying only in the concentration of the palmitate-albumin complex. The sequence of perfusion with buffers with different palmitate-albumin complex concentrations was in 5 out of 9 cardiac preparations from low to high, in the other 4 preparations the sequence was at random. The ratio of palmitate and albumin concentration was kept constant at 0.91. The choice of this ratio is rather arbitrarily, but corresponds with plasma *Fa*/*Alb* ratios commonly observed in humans and experimental animals [2].

The actual [*Alb*] studied was 0.0147 (8), 0.055 (9), 0.165 (6), 0.44 (7), 0.55 (2) and 0.88 (2) mmol l^-1^, with the number of experiments within brackets.

Indicator dilution curves were obtained by insertion of injectates into the flowing corresponding buffer-solution. The injectates, containing the radio-labeled tracers, possessed exactly the same chemical composition as the corresponding buffer-solutions, but a fraction of albumin and palmitate was replaced by their radio-labeled isoforms ^131^I-albumin (3 μCi) and ^14^C-palmitate (5 μCi), respectively. The ^131^I-albumin serves as to define transport through the intravascular compartment.

The buffer-solutions were kept in two-liter flasks in a temperature controlled water bath. With the use of various sets of pumps and distribution valves these oxygenated palmitate-albumin containing solutions were pumped through four parallel 8.5 μm filters, an in-line stainless steel heat exchanger, a water-jacketed Windkessel (to decrease pulsation and promote constant flow) and the injection valve into the aortic cannula to which the heart was connected. After the initial 10-min perfusion with the KRB-solution, the heart was perfused with the first of four albumin-containing solutions. After a 10 min equilibrium period, 1 ml of the corresponding injectate, containing radiolabeled albumin and palmitate, was inserted into the stream of perfusion solution just above the aorta cannula, to obtain the first set of indicator dilution outflow data points. Five minutes after injection of the radiolabeled tracers, the perfusate was switched to the second palmitate-albumin solution. Ten minutes later an aliquot of the second, corresponding injectate was inserted to obtain the second set of indicator dilution data points. The same procedure was followed to obtain the third and fourth set of data points, resulting in a total perfusion time of each heart of about 70 min. A 10 minutes equilibrium period was chosen as Tschubar and colleagues [7] found that in the isolated perfused heart equilibrium between the arterial and the interstitial albumin concentration was reached within 10 minutes.

The switch from perfusion with radiolabeled material to the next buffer without radiolabeled palmitate-albumin was performed after 5 minutes since pilot studies showed that after 5 minutes no measurable amounts of radiolabeled material could be detected in the coronary outflow samples. At the end of the last experiment any adherent lung and adipose tissue was removed carefully and the wet weights of the total heart and of the ventricles were measured.

### Sample collection and preparation, and radioisotope counting

To obtain the sets of data points mentioned above, coronary perfusate samples were collected from coronary sinus outflow into the right ventricle at intervals of one second for the first 30 samples making use of a small catheter inserted into the right ventricle apex and a custom-made fraction collector. Thereafter, an additional set of 30 samples was collected at four-second intervals. Collection of samples in glass test tubes was started routinely five seconds prior to injection of the injectate with radiolabeled tracers. The precision of the motor-driven fraction collector was tested in a pilot study. A volume of 0.1 ml of each outflow sample, and each standard and background sample, was pipetted into glass minivials. Ten microliter of glacial acetic acid was added to allow any ^14^CO_2_ present to escape. Then, a volume of 3 ml of Aquasol (New England Nuclear) was added and the mini-vial was vigorously shaken. Counting was performed in a liquid scintillation counter (Beckman Instruments). In order to assess correctly the ^14^C and ^131^I-counts, two sets of quench-spillover correction curves (^14^C and ^131^I), of 15 to 25 data points each, were made for each experiment. The experimental outflow data, expressed as counts per minute per sample point of each multiple indicator dilution experiment, was digitally stored for further processing (see below: “*Data storage and analysis”*).

### Preparation of perfusion solutions and injectates

#### Perfusion solutions

The KRB-buffer solution consisted (KRB-A) of (in mmol l^-1^) Na^+^ (143.0), K^+^ (5.0), Ca^2+^ (2.1), Mg^2+^ (0.7), Cl^-^ (124.0), HCO_3_^-^ (25.0), SO_4_^2-^ (0.7), HPO_4_^2-^ (1.2), EDTA^4-^ (0.1) and glucose (11.0), pH 7.4. The palmitate-albumin containing modified KRB-solutions were prepared as follows. First, the modified KRB-solutions containing appropriate concentrations of bovine serum albumin (BSA) were prepared. These solutions were dialyzed against the exchange KRB-A buffer using dialysis bags at 20°C for 5 hours to remove possible impurities in BSA used. Thereafter, the potassium-palmitic acid salts were added. The potassium-palmitate salts were made by dissolving appropriate amounts of palmitic acid in 1 ml 100% ethanol. K_2_CO_3_ (0.69 g dissolved in 5 ml H_2_O) was slowly added to the palmitic acid solution followed by stirring and gentle heating to 35°C. The solutions containing the palmitate-albumin complex were dialyzed overnight against a modified exchange KRB-A buffer using dialysis bags at 4°C to remove excess potassium ions. The final electrolyte composition of the palmitate-albumin solutions was (in mmol l^-1^): Na^+^ (143.0), Ca^2+^ (2.1), Mg^2+^ (0.7), K^+^ (5.0), Cl^-^ (124.0), SO_4_^2-^ (0.7), PO_4_^3-^ (1.2), HCO_3_^-^ (23.2), CO_3_^2-^ (0.5) and EDTA^4-^ (0.1). The final glucose concentration was 5.5 mmol l^-1^.

### Preparation of the injectates

For routine experiments (n = 34), the following two radiotracers were used:

- ^131^I-human serum albumin. Any fatty acid bound to ^131^I-albumin was removed by treatment with charcoal. Subsequently, to remove such impurities as free ^131^I (in the order of 1%) and aggregated albumin (about 0.1%), the ^131^I-albumin solution was dialyzed against distilled water with the use of a Spectra/por dialysis membrane at 4°C against 1 liter H_2_O for 12 hours. Thereafter, the dialysate was filtered through a 0.2 μm Nucleopore filter, using vacuum to remove any aggregates.
- Radio-labeled ^14^C-palmitic acid was tested for purity by silica gel thin-layer chromatography using petroleum ether/ diethyl ether/ acetic acid (80/20/1 by vol.) as a solvent system. Radiochemical purity of palmitic acid exceeded 99%. Before preparation of the injectates, the labeled palmitic acid was dissolved in 100 μl 100% ethanol. The major part of ethanol was removed by a gentle stream of N_2_. An appropriate amount of K_2_CO_3_ was dissolved in 250 μl H_2_O to obtain a final molar ratio of potassium: palmitate of 10:1. The K_2_CO_3_ solution was added and the resulting potassium-palmitate salt was dissolved under continuous stirring.

As the injectate, consisting of the radiolabeled albumin and palmitate tracers, is inserted into the stream of the solution flowing to the heart, the non-tracer concentrations of albumin, palmitate, salts and glucose of the injectate should perfectly match the concentrations in the corresponding perfusion solution. To this end, for each cardiac preparation four individual injectate solutions were carefully prepared. Based upon the specific activities of the ^131^I-albumin and ^14^C-palmitate, the desired amount of radioactivity (about 3 μCi ^131^I and 5 μCi ^14^C, respectively) and the final concentrations of albumin and palmitate in the injectate, the amounts of non-labeled BSA and palmitate to be added, were calculated. A 10% solution of BSA was filtered through a 0.2 μm Nucleopore filter. An aliquot of the filtered solution was added to the radiolabeled albumin solution to achieve the desired final concentration of albumin. The radioactive potassium-palmitate (about 5 μCi ^14^C) and an aliquot of a 0.5% non-radioactive potassium-palmitate solution were mixed and added to the albumin solution. Subsequently, salts, EDTA and finally NaHCO_3_ were added to the albumin-palmitate mixture to obtain a solution containing (in mmol l^-1^) Na^+^ (143.0), Ca^2+^ (2.1), Mg^2+^ (0.7), K^+^ (5.0), C1^-^ (124.0), SO_4_^2-^ (0.7), PO_4_^3-^ (1.2), HCO_3_^-^ (23.8), CO_3_^2-^ (0.5) and EDTA^4-^ (0.1). To substantially lower the CO_3_^2-^ concentration, to remove possible impurities present in the albumin solution and to add glucose, this mixture with a volume of 2.5 ml was dialyzed making use of a dialysis bag against 5.6 ml of (in mmol l^-1^) Na^+^ (143.0), Ca^2+^ (2.1), Mg^2+^ (0.7), K^+^ (5.0), C1^-^ (124.0), SO_4_^2-^ (0.7), PO_4_^3-^ (1.2), HCO_3_^-^ (24.2) and EDTA^4-^ (0.1) and glucose (7.3) at 4°C overnight in order to obtain an injectate solution with identical chemical composition as the corresponding non-radiolabeled perfusion solution. The dialyzing medium was gassed with 95% O_2_-5% CO_2_ at 36.5°C for 2h before the experiment. Prior to insertion, small aliquots of the injectate were taken to measure the radioactivity of the two tracers in the injectate, which provide a measurement of the injected dose.

### Chemicals and materials

Bovine serum albumin (BSA), essentially fatty acid free (A-7030), and palmitic acid (P-0500) were obtained from Sigma (St. Louis, MO, USA). ^14^C-Palmitic acid (850 mCi mmol^-1^) (uniformly labeled), dissolved in ethanol, was obtained from Amersham. ^131^I-Human serum albumin (750 mCi mmol^-1^), dissolved in 0.1 mmol l^-1^ phosphate buffer (pH 7.4), manufactured by Squibb, Inc., was obtained through Northwest Radio-pharmaceutical Services, Inc. All other chemicals were of reagent grade and purchased from Baker Chemical Co.

Dialysis bags were made from Spectra/por dialysis membrane (molecular weight cutoff: 12000–14000). The 0.2 μm membrane filters (mixed esters of cellulose acetate and cellulose nitrate) were obtained from Nucleopore, and 8.5 μm membrane filters (mixed esters of cellulose acetate and cellulose nitrate) from Millipore.

### Data storage and analysis

#### Data storage

Data from the multiple indicator dilution experiments, used in the present study, are stored in digital format. The related files ’AlbPalmVanDerVusse.zip’ are accessible through website: https://osf.io/tf2yd.

For each experiment the following data were obtained from the related file: coronary flow [ml s^-1^], ventricular mass [g], albumin and palmitate concentrations [mol m^-3^, *i*.*e*., mM], and sampled dilution curves (sampling times [s], initially normalized labeled albumin (*Alb*^*L*^) and palmitate (*Fa*^*L*^) concentrations [s^-1^]). Initial normalization of the albumin and fatty acids outflow curves was performed as described earlier [8].

### Data analysis

Per experiment, venous outflow samples were obtained as a function of time, allowing construction of labeled albumin and palmitate washout curves. Since albumin does not leave the coronary vessel compartment during the short time radiolabeled albumin and palmitate pass the capillaries, the albumin washout curve provides information about transport of compounds from coronary arteries to coronary veins without exchange with the myocardium. *Fa* are assumed to be exchanged only within the coronary capillary compartment and to be partially metabolized solely in the cardiomyocytes. Careful analysis of the difference between the albumin and *Fa* washout curves enabled us to retrieve relevant information about intra-cardiac *Fa* exchange and extraction. *Fa* exchange being defined as *Fa* taken up by and released from the tissue surrounding the microvascular compartment; *Fa* extraction as that part of the *Fa* taken up and not released back into the microvascular compartment due to metabolic conversion and long-term storage in the tissue, *i*.*e*., storage longer than the duration of the experimental sampling period.

Fig 2 schematically shows the sequence of calculations. Given coronary flow (experiment) and the physical properties of the coronary capillary compartment [9], the capillary impulse response function *H*(*t*) is calculated, following the procedure as described by Arts and coworkers [5]. The capillary impulse response function of a tracer is defined as the concentration at the exit of the capillary system as a function of time, assuming an infinitely short bolus injection of the tracer at the entrance of the capillary system.

**Fig 2:** Flow diagram of calculations carried out for the analysis. [*Alb*^*L*^] and [*Fa*^*L*^] refer to the total sample concentrations of labeled albumin, *Alb*^*L*^, and labeled palmitate, *Fa*^*L*^, *i*.*e*., free and bound combined, respectively. Data in the shaded upper left box, which are used as input, refer to experimental data. The resulting parameter value, shown in the shaded lower right box represents the output of the analysis. For the given coronary flow and the sampled washout curves for labeled *Alb*^*L*^ and *Fa*^*L*^, the most optimal fit between the experimentally obtained and simulated *Fa*^*L*^ washout samples was determined (see text for details); cap. refers to capillary.

Initially, normalized washout curves of labeled albumin, *Alb*^*L*^(*t*), and palmitate, *Fa*^*L*^(*t*), were derived from the time sequence of experimentally obtained samples of labeled *Alb*^*L*^ and *Fa*^*L*^ concentrations, measured at the outlet of the coronary system [10]. In the present analysis, the outflow curves *Alb*^*L*^*(t)* and *Fa*^*L*^*(t)* are represented as continuous functions obtained by interpolation of the related sample points in the measuring interval and attachment of the tail by extrapolation (details are described in Appendix 1). Finally, the total time integral of *Alb*^*L*^*(t)* was set equal to 1.0 by multiplication with an appropriate normalization factor. The outflow curve *Fa*^*L*^*(t)* was obtained by multiplication with the same normalization factor.

*Fa* extraction was determined as the difference between the time integral of the radiolabeled *Alb* curve, which was set equal to 1.0, and the time integral of the radiolabeled *Fa* curve. In a small number of experiments, the thus found extraction appeared to be negative, which is physically impossible because the heart cannot produce radioactively labeled *Fa*. We attributed this anomaly to inaccuracies in the radioactivity measurements. Assuming that the error in the assessment of the time integral is distributed normally, we determined the most likely value for the true extraction, taking into account that labeled *Fa* extraction could not be negative. The correction was carried out by multiplying the measured [*Fa*^*L*^](*t*) curve with a correction factor so that *Fa* extraction was equal to the most likely value determined in this correction procedure. Details thereof are described in Appendix 2. For 6 out of 34 curves, the correction was more than 1%. For this group of 6, the average correction was 2.8±0.8% (mean±sd).

The next step was to obtain the simulated *Fa*^*L*^ curve by means of our model as described in detail previously [5]. To sum up, we obtained the curve [*Alb*^*L*^]_*dec*_(*t*) by deconvolution of the measured dilution curve [*Alb*^*L*^](*t*) with the simulated capillary impulse response curve *H*(*t*). The deconvoluted curve [*Alb*^*L*^]_*dec*_(*t*) represents the *Alb* dilution curve of the combined arterial and venous parts of the total coronary system, without the capillary section. Since we assume that exchange of *Fa* solely occurs in the capillary section of the coronary system, the deconvoluted *Fa* curve, [*Fa*^*L*^]_*dec*_(*t*), *i*.*e*., the coronary *Fa* dilution curve without the contribution of the capillaries, was set equal to [*Alb*^*L*^]_*dec*_(*t*). Subsequently, the curve [*Fa*^*L*^]_*dec*_(*t*) was used as input to that part of the model dealing with the *Fa* transfer in the capillaries, *i*.*e*., *Fa* exchange and extraction within the cardiac tissue, yielding the simulated *Fa* dilution curve [*Fa*^*L*^]_*sim*_(*t*).

Simulation of cardiac *Fa* exchange and extraction requires the values of a specific number of parameters. Some of these values are available from experimental data published in literature (Tables 1 and 2). However, the values of three parameters, considered to be essential for transfer of *Fa* from the capillary compartment through the endothelium to the cardiomyocyte, are to be estimated from our experimental data. As already indicated in the introduction, these three parameters are: i) the dissociation time constant of the *AlbFa* complex, *τ*_*AlbFa*_, ii) the membrane reaction rate parameter, *d*_*Alb*_ and iii) *Fa* permeability of the endothelial cytoplasm, *P*_*ec*_. Both *τ*_*AlbFa*_ and *d*_*Alb*_ are parameters relevant for three extracellular membrane interfaces, *i*.*e*., the capillary-endothelial, the endothelial-interstitial and the interstitial-cardiomyocyte interface.

**Table 1:** Physics-related parameters.

Variable	Unit	Value	Reference
Diffusion constant			
Albumin	m^2^ s^-1^	9.35∙10^−11^	[32]
Palmitate	m^2^ s^-1^	4.4∙10^−10^	[32, 33]
Molecular mass			
Albumin	D	67000	[34]
Palmitate	D	256	
Partition coefficient *Fa* (membrane/water)	-	8∙10^5^	[35]
Cardiac tissue density	kg m^-3^	1050	https://bionumbers.hms.harvard.edu/files/Density%20and%20mass%20of%20each%20organ-tissue.pdf
Membrane thickness	nm	5	[36]
Capillary diameter	μm	5.2	[9]

**Table 2:** Compartment-related parameters.

Variable	Unit	*cap* ^a)^	*ec* ^a)^	*is* ^a)^	*myo* ^a)^
Volume fraction ^b)^	‰	94	18	19+60^c)^	731
Diffusion thickness ^d)^	nm	762	NR	160	NR
*Cp*, molecule type	-	Alb	FABP_ec_	Alb	FABP_myo_
Equilibrium constant *CpFa*	mol m^-3^	8.5∙10^−6 e)^	like myo	like cap	4∙10^−6 e)^
Dissociation time	ms	fit	NR	like cap	NR
Contact pathway *d*_*Cp*_	nm	2/20/200	NR	like cap	NR
Concentration [*Cp*]	mol m^-3^	^f)^	like myo	85% of cap^h)^	0.17 ^j)^
Membrane area/tissue volume ^k)^	m^2^ m^-3^	75200	89000	94000	

a) *cap*, *ec*, *is*, *myo* refer to capillary, endothelial, interstitial and cardiomyocytal compartments, respectively.

b) Data obtained from [9]. The remaining volume (78‰) represents large blood vessels and other cells types.

c) Interstitium between endothelium and cardiomyocyte, and interstitium between cardiomyocytes, respectively.

d) Data obtained from [9]. Note that for a capillary diameter of 5.2 μm, the median diffusion distance between endothelial luminal membrane and the capillary fluid content is 762 nm.

e) Obtained from [22, 37].

f) Varies per experiment.

h) Obtained from [7].

j) Obtained from [38].

k) Surface area of the luminal endothelial membrane, abluminal endothelial membrane and sarcolemma per unit tissue volume, respectively. Data obtained from [9].

NR: not relevant for present analysis.

Next, the model data points were fitted with the experimental data points by variation of *τ*_*AlbFa*_, so that the difference between simulated and measured radiolabeled *Fa* concentrations in the samples was minimal. The latter difference was quantified by an objective function as described in detail in Appendix 3. For all 34 multiple dilution experiments, the fits were carried out with input variables *d*_*Alb*_ and *P*_*ec*_ in the following combinations (units: nm and mm s^-1^, respectively): [2, 200], [20, 200], [200, 200], [20, 50], which was a wide range, considered to cover the most likely values of these parameters in cardiac *Fa*-transfer. The unit nm of the membrane reaction rate parameter, *d*_*Alb*_, stems from Eq 24 of the mathematical model published in detail in [5]. The membrane reaction rate parameter, *d*_*Alb*_, represents the actual thickness (in nm) of the boundary zone with aberrant concentrations of *Fa*-free albumin due to the direct transfer of *Fa* from the complex into the cell membrane. The disturbance in the equilibrium of *Fa*-free albumin and the *AlbFa* complex is restored by diffusion of *AlbFa* complex molecules from the bulk. If the efficacy of direct transfer of *Fa* from *AlbFa* complex into the membrane increases, the thickness of the layer (in nm) in the boundary zone with disturbed equilibrium between *Fa*-loaded and *Fa*-free albumin increases as well, which implies an increase of the value of *d*_*Alb*_ (also with unit nm).

In the fitting procedure, total *Fa*-permeability from capillary to cardiomyocyte, *P*_*tot*_, for each experiment was calculated as the in-series combination of the permeabilities of the capillary, endothelial, interstitial and cardiomyocyte compartments and all related cell membranes, having boundary zones on both sides, to be crossed. Details of the calculation procedure of *P*_*tot*_ have been published previously by Arts and coworkers [5]. To sum up, we applied the rule that the total permeability of individual permeabilities in series, *P*_*tot*_, equals the reciprocal of the sum of reciprocals of these individual permeabilities. In this procedure, the values of the boundary zone inside the cardiomyocyte and endothelial cell were assumed to be similar. Moreover, since previous calculations revealed that *Fa* permeability of a phospholipid bilayer is very high [5], the permeabilities of the three cell membranes to be crossed were considered to be inconsequential in the assessment of total cardiac permeability, *P*_*tot*_, and could, therefore, be neglected.

The overall conductance of the serial processes, *P*_*tot*_, is essential for understanding the impact of the individual steps on overall *Fa*-hindrance in their transfer from capillary to interior of the cardiomyocyte. Therefore, we performed a linear regression analysis on the logarithm of *P*_*tot*_ as a function of the logarithm of the total capillary albumin concentration, [*Alb*], yielding the mean value ± SEM of the slope of log*P*_*tot*_/log[*Alb*] for the 34 experiments. The rationale behind this regression analysis is based upon previous findings in our model of intra-cardiac *Fa* exchange indicating that *P*_*tot*_ increases with increasing [*Alb*] [5]. The slope of the regression line of the relationship between *P*_*tot*_ and [*Alb*] is determined by the combined effect of all compartments to be crossed in intra-cardiac *Fa*-transfer [5]. Therefore, analysis of the relationship between *P*_*tot*_ and [*Alb*] found experimentally provides important information regarding which sites are dominating the total cardiac *Fa* permeability, *P*_*tot*_.

As the values of the three, most relevant parameters are largely unknown, *i*.*e*., for *d*_*Alb*_ and *P*_*ec*_ no accurate data are available at all, while the values published for *τ*_*AlbFa*_ show substantial variation, we decided to estimate the most likely range of the values of [*τ*_*AlbFa*_, *d*_*Alb*_]. Likelihood was estimated on the basis of theoretical and experimental considerations: *P*_*ec*_ should not become negative and the slope of estimated log*P*_*tot*_*/*log*[Alb]* should be within the range ±2 SEM around the experimentally obtained mean value. To make the estimation procedure manageable, after performing regression analysis on the experimentally obtained plot of *Y* = ^10^log(*P*_*tot*_) versus *X* = ^10^log([*Alb*]), we focused on the center of gravity [*X*_*M*_, *Y*_*M*_] of all data points in the plot because the relationship between *Y* and *X* is most accurately known around this center of gravity. It is of note that, by applying linearity of the relation between *X* and *Y*, the center of gravity is located on the regression line. Furthermore, the derivative d*Y*/d*X* in the center of gravity corresponds with the slope *m* of the regression line, as discussed above. In further analysis of *P*_*tot*_ as a function of [*Alb*], the *Fa* extraction fraction was set at 0.1, corresponding with the median value of the extraction fractions found experimentally. The center of gravity [*X*_*M*_, *Y*_M_] obtained experimentally corresponds with the values *P*_*tot*,*Mexp*_ and [*Alb*]_*Mexp*_.

Using the *Fa* exchange model [5] with the given [*Alb*], the value of *P*_*tot*_ is described as a function of *d*_*Alb*_, *τ*_*AlbFa*_, and *P*_*ec*_. In our subsequent analysis, variables *d*_*Alb*_ and *τ*_*AlbFa*_ ranged from 5 to 500 nm and from 0.05 to 5.0 s, respectively, both sampled in 40 logarithmically equidistant steps. Thus, for *P*_*tot*,*Mexp*_, we solved *P*_*ec*_ numerically as a function of *d*_*Alb*_, *τ*_*AlbFa*_ for all 1600 combinations of *d*_*Alb*_ and *τ*_*AlbFa*_ (Fig 3, left panel). Next, with the same *Fa* exchange model, for each triplet of *d*_*Alb*_, *τ*_*AlbFa*_, and *P*_*ec*_ values we calculated the slope *m* of the relation *Y*_*sim*_(*X*) around the point [*X*_*M*_,*Y*_*M*_] (Fig 3, right panel) applying

$$m=\frac{Y_{sim}(X_{M}+\Delta X)-Y_{sim}(X_{M}-\Delta X)}{2\Delta X}\;with\;\Delta X=0.5$$ (1)

**Fig 3:** Schematic representation of the estimation of *P*_*ec*_ as function of *d*_*Alb*_ and *τ*_*AlbFa*_ using the mathematical model published in Arts *et al*. [5] (left panel). The values of the input-variables *d*_*Alb*_ and *τ*_*AlbFa*_ varied from 5 to 500 [nm] and from 0.05 to 5.0 [s] in 40 logarithmically equidistant steps, respectively, yielding 1600 combinations of [*d*_*Alb*_,*τ*_*AlbFa*_]. The value of the third input-variable *P*_*ec*_, was adjusted so that the simulated value of total permeability in the center of gravity, ^10^log(*P*_*totM*,*sim*_), was equal to the experimentally determined value of ^10^log(*P*_*totM*,*exp*_) in the center of gravity. For calculating ^10^log(*P*_*totM*,*exp*_), the values of the gradients of free [*Fa*] between and within the various compartments are required. These values were derived from the *Fa* extraction fraction determined in the experiments. For the center of gravity, the *Fa* extraction fraction was set at 0.1. The right panel elucidates the calculation of slope *m* of the regression line (Eq 1), given the values of *d*_*Alb*_ and *τ*_*AlbFa*,_ and the value of *P*_*ec*_ as obtained from the calculation in the left panel. For all 1600 combinations *[d*_*Alb*_, *τ*_*AlbFa*_*]*, *P*_*ec*_ and *m* were calculated for further analysis.

Since *P*_*ec*_ is a function of *d*_*Alb*_ and *τ*_*AlbFa*_, we obtained 1600 *m*-values for all combinations of *d*_*Alb*_ and *τ*_*AlbFa*_. For graphical purposes, we also calculated *P*_*ec*_ and slope *m* for all 40 values of *τ*_*AlbFa*_ in combination with *d*_*Alb*_ approaching zero.

To estimate the relative contributions of the contact and the detach pathway to the overall *Fa*-flux from capillary to the cardiomyocyte in the boundary compartments containing albumin, we used Eq (6) reported previously in Arts and colleagues [5]. This equation indicates that the decay distance constant, *d*_*Fa*_, is more appropriate to quantify the detach pathway than *τ*_*AlbFa*_ because of the dependency of *d*_*Fa*_ on more relevant parameters involved, such as [*Alb*_*free*_] as shown in Eq 2 below. From Eq 6 (5) we derived that the ratio of contact pathway flux *φ*_*c*_ to detach pathway flux *φ*_*d*_ equals:

$$\frac{\varphi_{c}}{\varphi_{d}}=\frac{d_{Alb}}{d_{Fa}}\;\mathrm{with}\;d_{Fa}=\sqrt[{}]{\frac{D_{Fa}K_{AlbFa}\tau_{AlbFa}}{\left[{Alb}_{free}\right]}}$$ (2)

Parameters *D*_*Fa*_, *K*_*AlbFa*_, *τ*_*AlbFa*_ and [*Alb*_*free*_] indicate *Fa*-diffusion coefficient, *AlbFa* equilibrium constant, *AlbFa* dissociation time constant and the concentration of available albumin high-affinity *Fa* binding sites, respectively. We assumed that each albumin molecule contains 3 high-affinity *Fa* binding sites (3). From Eq (2) it follows that the relative contribution of the contact pathway to the total *Fa* flux in the boundary zone equals *d*_*Alb*_*/(d*_*Alb*_*+d*_*Fa*_*)* x100%. Likewise, *d*_*Fa*_/(*d*_*Alb*_*+d*_*Fa*_*)* x 100% represents the relative contribution of the detach pathway.

### Statistical analysis

Statistical analysis was performed by standard linear regression analysis. P<0.05 was considered statistically significant.

## Results

In the left panel of Fig 4, the net extraction fraction of labeled *Fa* by the myocardium is shown to be 34%±7% (mean ± sd) at 0.0147 mol m^-3^ [*Alb*] in the perfusate. The net extraction fraction dropped to 4%±3% at the highest range of [*Alb*] investigated, *i*.*e*., 0.44 to 0.88 mol m^-3^. While the net extraction fraction declined significantly, the total amount of *Fa* extracted increased significantly with increasing [*Alb*] (Fig 4, right panel).

**Fig 4:** Left panel: Experimentally determined net extraction fraction of labeled *Fa* by the isolated rabbit heart as function of total [*Alb*] in the perfusate (see Methods for actual albumin concentrations used). The net *Fa* extraction fraction [–] declines significantly with increasing albumin concentration (linear regression analysis, P<0.001). Right panel: Total amount of *Fa* extracted [nmol g^-1^ min^-1^] as function of total [*Alb*] in the perfusate. Extraction for each individual experiment was calculated by multiplying the net extraction fraction with flow [ml g^-1^ min^-1^] and the total concentration of *Fa* in the perfusate [mol m^-3^]. Extraction increased significantly with total [*Alb*] (P<0.01). The grey vertical line perpendicular on the x-axis indicates the physiological capillary albumin concentration, *[Alb]* = 0.64 mol m^-3^ [16].

Fig 5 shows four representative examples of simulated [*Alb*^*L*^] and [*Fa*^*L*^] outflow curves and corresponding experimentally obtained data points. The related [*Alb*^*L*^]_dec_ and [*Fa*^*L*^]_dec_ inflow curves obtained by deconvolution are shown as well. In these four examples, perfusate [*Alb*] amounted to 0.0147, 0.055, 0.165, 0.44 mol m^-3^ (= mmol l^-1^), respectively. The four examples show a good fit between model and experiment.

**Fig 5:** Four examples of simulated [*Alb*^*L*^] and [*Fa*^*L*^] outflow curves and corresponding data points determined experimentally. The related [*Alb*^*L*^]_*dec*_ and [*Fa*^*L*^]_*dec*_ inflow curves calculated are drawn as well. In these four examples, total perfusate [*Alb*] amounted to 0.0147, 0.055, 0.165 and 0.44 mol m^-3^; the ratio of perfusate total [*Fa*] over total [*Alb*] was 0.91. The fitting procedure was performed for values of the input variables *d*_*Alb*_ and *P*_*ec*_ set at [2,200] in [nm, mm s^-1^].

The relation between total cardiac *Fa*-permeability, *P*_*tot*_, and the capillary albumin concentration, [*Alb*], in the 34 multiple indicator dilution experiments is shown in Fig 6. Plotting *Y =* ^*10*^log*(P*_*tot*_*)* as a function of *X =* ^*10*^log*([Alb])* and applying linear regression analysis to the data points, a significant linear relation was found between *P*_*tot*_ and total [*Alb*], both plotted on a logarithmic scale.

**Fig 6:** The logarithm of total *Fa* permeability, *Y* = ^10^log(*P*_*tot*_), as a function of the logarithm of [*Alb*], *X* = ^10^log([*Alb*]), for all 34 experiments (see methods for actual albumin concentrations used). Each data point in the Fig represents the mean ± SD of *P*_*tot*_ values of the four combinations of [*d*_*Alb*_, *P*_*ec*_] examined (see Methods). Linear regression analysis with *Y*-*Y*_*M*_ = *m*(*X*-*X*_*M*_) yielded *X*_*M*_ = −1.00, *Y*_*M*_ = 0.365±0.032 and slope *m* = 0.49±0.05 (mean ± SEM) (P<0.001). Point *M* on the regression line represents the center of gravity, [*X*_*M*_,*Y*_*M*_], of all data points obtained experimentally. Point *Ph* refers to the physiological [*Alb*] = 0.64 mol m^-3^ in blood plasma [16]. [*X*_*Ph*_,*Y*_*Ph*_] = [-0.155, 0.777] implying *P*_*tot*_ = 5.98 mm s^-1^ at physiological [*Alb*]. Linear regression analysis of the slope of data points with flow values above the median vs. data points below the median value for a given [*Alb*] showed no significant effect of flow on the relation between *P*_*tot*_ and [*Alb*] (P>0.05).

It is of note that for each individual experiment, calculated *P*_*tot*_ varied only about 1.5% (Standard Deviation) for all four combinations of *d*_*Alb*_ and *P*_*ec*_ that were investigated and the related *τ*_*AlbFa*_ found in the fitting procedure. This implies that *P*_*tot*_ can be estimated reliably for each experimental condition, despite the fact that at this stage the physiologically correct values of *d*_*Alb*_ and *P*_*ec*_ are not known. The relationship in Fig 6 shows that the center of gravity *M* of all 34 experimental data points, [*X*_*M*_,*Y*_*M*_], equals [-1.00, 0.365], corresponding with [*Alb*]_*M*_ = 0.1 mol m^-3^ and *P*_*totMexp*_ = 2.32 mm s^-1^. The mean value and SEM of slope *m* of the regression line of *Y* as a function of *X* determined experimentally was 0.49±0.05 (linear regression analysis, P<0.001).

Fig 7A shows the values of *P*_*ec*_, calculated as a function of each of the 1600 combinations of the two variables *d*_*Alb*_ and *τ*_*AlbFa*_ as explained schematically in Fig 3. Subsequently, we plotted the *P*_*ec*_ level contour lines in the plane spanned by *d*_*Alb*_ and *τ*_*AlbFa*_ in horizontal and vertical direction, respectively. For the [*d*_*Alb*_,*τ*_*AlbFa*_] combinations in area E1, the calculated value of *P*_*ec*_ appeared to be negative, which is physically impossible. This makes the combinations of [*d*_*Alb*_, *τ*_*AlbFa*_] in region E1 unrealistic and, hence, should be discarded. Fig 7B shows the slope *m* = d*Y*/d*X*, calculated as the derivative of the logarithm of total permeability, *P*_*tot*_, with respect to the logarithm of [*Alb*] according to Eq (1) as shown in the Method section. Slope *m* was plotted as a function of the two variables *d*_*Alb*_ and *τ*_*AlbFa*_. Subsequently, we drew the level contour lines through the values of slope *m* in the plane spanned by *d*_*Alb*_ and *τ*_*AlbFa*_ in horizontal and vertical direction, respectively. The combinations of the variables *d*_*Alb*_ and *τ*_*AlbFa*_ in area E1 must be discarded as indicated in Fig 7A. For the [*d*_*Alb*_,*τ*_*AlbFa*_] combinations in area E2 in panel B, the value of slope *m*, calculated with the model, appeared to be to be more than 2 SEM distant from the mean value of slope m of the regression line found experimentally. Therefore, the combinations of *d*_*Alb*_ and *τ*_*AlbFa*_ in area E2 must be discarded as well. All [*d*_*Alb*_,*τ*_*AlbFa*_] combinations, yielding values of slope *m* higher than two times SEM lie within area E1 and, therefore, are not shown separately in Fig 7B. Combining panel A and B of Fig 7 results in panel C. As indicated, all [*d*_*Alb*_,*τ*_*AlbFa*_] combinations in both areas E1 and E2 are unlikely, leaving a narrow white band of acceptable [*d*_*Alb*_,*τ*_*AlbFa*_] and related *P*_*ec*_ values.

**Fig 7:** Panel A shows the level contour lines of *P*_*ec*_, as function of *d*_*Alb*_ and *τ*_*AlbFa*_. The line indicated with ∞ refers to infinite endothelial *Fa* permeability *(i*.*e*., zero endothelial hindrance of *Fa* diffusion). The combinations of [*d*_*Alb*_, *τ*_*AlbFa*_] in the gray area E1 are unlikely as it is physically impossible that *P*_*ec*_ is negative. The narrow vertical band at the left end site of the Fig reflects the situation for *d*_*Alb*_ approaching zero. Panel B shows the level contour lines of the slope value *m* = d*Y*/*dX*, calculated as the derivative of the logarithm of total permeability, *P*_*tot*_, with respect to the logarithm of [*Alb*] (see Fig 6), as a function of τ_*AlbFa*_ and *d*_*Alb*_. The bold contour line and white band represent, respectively, the mean ± 2SEM of the slope values found experimentally as shown in Fig 6, *i*.*e*., 0.49±2x0.05. As indicated in panel A, the combinations of [*d*_*Alb*_, *τ*_*AlbFa*_] in the gray area E1 are unlikely. Therefore, the bold line lying in area E1 is indicated as a broken line. The combinations of [*d*_*Alb*_, *τ*_*AlbFa*_] in the gray area E2 are unlikely for statistical reasons, since in that region the value of slope *m* differs more than 2 times SEM from the mean value found experimentally. In panel C the white band between the gray areas E1 and E2 represents values of *P*_*ec*_ as function of all acceptable combinations of [*d*_*Alb*_, *τ*_*AlbFa*_]. Panel C indicates that the lower limit of *P*_*ec*_ equals 7.5 mm s^-1^ with an upper limit approaching infinity.

By exclusion of the areas E1 and E2, Fig 7C indicates that, in case of *d*_*Alb*_ ≤5 nm, the true value of *τ*_*AlbFa*_ may vary between 0.2 and 0.4 s, with related values of *P*_*ec*_ varying from 15 mm s^-1^ to infinity. In case *d*_*Alb*_ is higher than 5 nm, at a given value of *τ*_*AlbFa*_, the estimated value of *P*_*ec*_ declines. If the true value of *τ*_*AlbFa*_ were higher as well, the value of *P*_*ec*_ might range from 7.5 mm s^-1^ unto infinity.

## Discussion

Blood-borne *Fa* are important substrates for the heart. Due to the very low solubility of *Fa* in water, *Fa*-binding proteins, such as albumin in the vascular and interstitial compartment and Fatty Acid-Binding Proteins, *FABP*, in the intracellular compartments, are required to facilitate the diffusional transfer of *Fa* from capillary to cardiomyocyte. In this trajectory, *Fa* must traverse a number of aqueous compartments such as the cytoplasm of the endothelial and cardiac muscle cells and fluid layers in the extracellular capillary and peri-vascular interstitium, and the lipophilic cell membranes, all potentially playing a decisive role in the resistance to *Fa* transfer in cardiac tissue. Moreover, the involvement of *Fa*-binding proteins in cardiac *Fa*-diffusion implies that *Fa* are not only delivered to cell membranes as free *Fa*, *i*.*e*., via the detach pathway, but also as protein-bound *Fa*, *i*.*e*., via the contact pathway [5]. Despite the quantitative importance of *Fa* for cardiac energy conversion, our knowledge of the processes underlying the transfer of *Fa* from capillary to cardiomyocyte is limited. In the present study, our aims were to delineate the site of highest hindrance of cardiac *Fa* diffusion (*i*.*e*., the site with the lowest *Fa* permeability) in the overall *Fa* diffusion trajectory, and the relative importance of the detach and the contact pathway in delivering *Fa* to the cellular membranes in the compartments containing albumin.

In our analyses, we used an extensive set of 34 multiple indicator dilution experiments performed on isolated rabbit hearts and a mathematical model published previously, dealing with intra-cardiac *Fa* transfer [5]. Indicator dilution experiments are the experimental model of choice to investigate the dynamic behavior of *Fa* exchange in the intact heart [10, 11]. The present approach allows for getting insight into the bidirectional transfer of labeled *Fa* in the heart during a single pass of the substrate in the coronary capillaries. Studies on isolated or cultured cells are not appropriate to investigate the dynamic behavior of cardiac *Fa* transfer since they lack the intricate relationship between the various compartments and cell types involved in cardiac *Fa* exchange and extraction, especially on seconds to minutes scales.

The strength of the present study is the application of a mathematical model published earlier which allows derivation of relevant physiological information from radiolabeled albumin and *Fa* coronary outflow curves obtained experimentally. This mathematical model is based upon standard physicochemical principles of diffusion, taking into account the chemical equilibrium of *Fa* binding to carrier proteins in the extra- and intracellular compartments. In this model, concentration differences of free *Fa* between and inside relevant aqueous compartments are the driving force of intra-cardiac *Fa* diffusion. The fact that the experimental findings could be very well fitted with the findings obtained with the mathematical model justifies the conclusion that in the intact heart intra-cardiac *Fa* transfer is accomplished by passive diffusion. Other mathematical models previously published which were designed to shed more light on cardiac *Fa* transfer either lacked discrimination between free *Fa* and *Fa* bound to carrier-proteins like albumin or *FABP* [6] or remain purely theoretical without analysis of experimental data [12–14].

Since we applied an isolated *ex vivo* perfused rabbit heart as experimental model to investigate cardiac *Fa* transfer, the question can be raised as to whether this experimental *ex vivo* model allows for extrapolation of the present findings to the intact heart *in situ*. Fig 4, right panel, shows that around the physiological [*Alb*] in plasma, *i*.*e*., 0.64 mol m^-3^, the total amount of *Fa* extracted is about 30 to 150 nmol g^-1^ min^-1^. This amount corresponds very well with the net consumption rate of *Fa* in the open-chest dog heart, ranging from 16 to 137 nmol g^-1^ min^-1^ [15], justifying the conclusion that the present experimental set-up provides relevant information for the physiological situation of the beating mammalian heart *in situ*.

To identify the site of lowest *Fa* permeability (highest *Fa* hindrance) in the diffusion pathway of *Fa* from capillary to cardiomyocyte, the *Fa* permeability of the total trajectory, *P*_*tot*_, has to be compared with the individual permeabilities of the constituting compartments and cellular membranes. In the diffusion trajectory of *Fa* from capillary to cardiomyocyte, eleven potential sites of hindrance are present. They are the bulk and boundary zone in the capillary containing albumin, the endothelial luminal membrane, two boundary zones inside the endothelial cell containing *FABP*_*ec*_, the abluminal endothelial membrane, two boundary zones in the peri-capillary interstitium containing albumin, the sarcolemma, and one boundary zone and bulk inside the cardiomyocyte containing *FABP*_*myo*_. Because of the narrow width of the endothelial cell and peri-capillary interstitium [9], in these anatomical compartments the two boundary zones merge into each other leaving no room for a bulk. Under physiological conditions, the concentrations of albumin and *FABP*_*myo*_ in the capillary and cardiomyocyte compartment, respectively, is relatively high [4, 16]. Therefore, when we calculated the summed effect of the related bulk *Fa-*permeabilities on *P*_*tot*_ using Eq, 8 in Arts *et al*. [5], this effect appeared to be less than 1% and, hence, negligible. Since the impact of membrane permeability on *P*_*tot*_ was also negligible [5], the conclusion is justified that the main sites of hindrance are the three albumin-containing extra-cellular boundary zones, one in the capillary and two boundary zones in the peri-capillary interstitium, and the three *FABP*-containing intra-cellular boundary zones, *i*.*e*., the two boundary zones in the cytoplasm of the endothelial and one in the cytoplasm of the cardiac muscle cell.

It is of note that endothelial permeability, *P*_*ec*,_ depends on the endothelial *FABP* concentration, [*FABP*_*ec*_], the dissociation constant, *k*_*d*_, for *Fa* binding to *FABP*_*ec*_, the *FABP*_*ec*_ dissociation time constant, *τ*_*FABPecFa*_, and the endothelial membrane reaction rate parameter (*d*_*FABPec*_). The latter parameter quantifies the importance of the endothelial *Fa* contact pathway, involving *Fa* transfer by physical contact of *FABP*_*ec*_ with the cytoplasmic side of the luminal and abluminal endothelial membrane, followed by direct translocation of *Fa*. At present, no information is available about the real values of endothelial *τ*_*FABPecFa*_, *k*_*d*_, and *d*_*FABPec*_. Moreover, the concentration of *FABP* in the endothelial cytoplasm reported in literature differs considerably among the various investigations [17–20]. The uncertainties in these parameter values prompted us to apply the overall parameter *P*_*ec*_ in estimating intra-endothelial *Fa*-permeability. Due to the narrow width of the endothelial cell, the endothelial cell permeability consists of two *FABP*_*ec*_-containing boundary zones merging into each other. With respect to the permeability of the intra-cardiomyocyte boundary zone, *P*_*b*,*myo*_, we assumed the values of the concentration of *FABP*_*myo*_, *τ*_*FABPmyoFa*_, and *d*_*FABPmyo*_ to be equal to those of endothelial *FABP*. Since the cardiomyocyte contains only one boundary zone instead of two, as in the endothelial cell, the value of *P*_*b*,*myo*_ is about two times higher than *P*_*ec*_.

In a seminal study, Rose and Goresky [6] concluded that the endothelium poses the greatest constraint to cardiac *Fa* uptake, but they did not take into account the contribution of albumin-delivered *Fa* to the endothelial cell membrane via the contact pathway. In contrast, Tschubar and colleagues [7] concluded that the endothelium could not play a significant role at all in cardiac diffusion resistance. They based their conclusion on measurement of the unbound *Fa* concentration in the interstitial fluid relative to the concentration in the capillary lumen. Moreover, they assumed the endothelial [*FABP*] to be sufficiently high for unimpeded *Fa* diffusion inside the endothelial cells. The present analysis of indicator dilution experiments, however, shows that we must be more cautious in considering a role of the endothelium in hindering *Fa* diffusion from capillary to cardiomyocyte. This conclusion is illustrated by the outcome of our analysis of physiologically acceptable values of [*τ*_*AlbFa*_, *d*_*Alb*_] as function of endothelial permeability, *P*_*ec*_ (Fig 7C). In case the true value of *τ*_*AlbFa*_ = 0.2 s, *P*_*ec*_ equals 15 mm s^-1^. At the physiological [*Alb*] of 0.64 mol m^-3^ [16], *P*_*tot*_ amounts to 5.98 mm s^-1^ (Fig 6) and, hence, the effect of the *Fa*-permeability of the endothelial cell interior, *P*_*ec*_, on *P*_*tot*_ is notable, *i*.*e*., about 40%. If the *Fa* dissociation from albumin is slower, *e*.*g*. *τ*_*AlbFa*_ = 400 ms, the permeability of the endothelial cytoplasm, *P*_*ec*_, may vary from infinite (no hindrance) to about 8.5 mm s^-1^ (high hindrance). It is of note that in case *P*_*ec*_ is approaching infinity, the main hindrance towards intra-cardiac *Fa* transfer must be located in the three albumin-containing boundary zones, one in the capillary and two merging into each other in the peri-capillary interstitium to keep the total intra-cardiac *Fa* flux at the level determined in the experiments.

Our study clearly shows that no definitive conclusion can be drawn regarding the contribution of the endothelial cytoplasm to the overall intra-cardiac resistance to *Fa* diffusion due to the lack of reliable experimental data regarding the value of *d*_*Alb*_ and the substantial variation in values of *τ*_*AlbFa*_, found in the literature, the latter varying from 0.14 s to over 60 s [21–24]. This variation mainly results from differences in experimental conditions and in interpretation of the experimental outcome. The present findings indicate that solid experimental data on the true *τ*_*AlbFa*_ and *d*_*Alb*_ are required to allow precise assessment of the impact of the endothelium on total cardiac *Fa* permeability.

Two parallel pathways, the contact and the detach pathway, determine *Fa*-permeability of the fluid in the boundary zones adjacent to the cell membranes. It is of note that the contact and the detach pathway are connected at the site where *Fa* translocate from the fluid layer in close vicinity to the cell membrane, either as free *Fa* (detach) or as *Fa* bound to a *Fa*-carrier protein, *Cp* (contact pathway). Eq 24 in Arts *et al*. (PLOS, 2015) shows that, in the case of absence of net transfer of *Fa* along the detach pathway, the free *Fa* concentration in the fluid bulk is in equilibrium with the much higher *Fa* concentration in the membrane. As total *Fa* flux from capillary to cardiomyocyte occurs via passive diffusion, *i*.*e*., a process that does not require external energy, the physical principle of conservation of energy dictates that this equilibrium also holds for the contact pathway.

In the extracellular boundary zones in the capillary as well as in the peri-vascular interstitium, albumin serves as *Fa*-carrier protein. The identification of the acceptable range of [*τ*_*AlbFa*,_ *d*_*Alb*_] (Fig 7C) enables us to estimate the relative contribution of the contact and detach pathways to the *Fa* flux in these boundary zones under physiological [*Alb*] conditions. To this end, we determined the ratio *d*_*Alb*_*/d*_*Fa*_ applying Eq (2) (Method section). In case the true value of *τ*_*AlbFa*_ equals 0.2 s with an accompanying value of *d*_*Alb*_ of maximally 5 nm (Fig 7C), the estimated contribution of the contact pathway amounts to maximally 20%. In case *τ*_*AlbFa*_ equals 0.4 s, the maximal value of *d*_*Alb*_ is about 100 nm. Under these conditions, the estimated contribution of the contact pathway will be considerably higher. As indicated above, the estimation of the precise contribution of the contact and detach pathway to permeability of the boundary zone is hampered because of the lack of information on the exact value of *d*_*Alb*_ and the uncertainty in the true value of *τ*_*AlbFa*_ reported in literature.

It should be realized that of the two parameters, *τ*_*AlbFa*_ and *d*_*Alb*_, determining the permeability of the boundary zones, *P*_*b*_, and, hence, *P*_*tot*_, the first one is a fixed material constant and, therefore, not subject to regulation on a short-term basis. The value of the membrane reaction rate parameter, *d*_*Alb*_, may be adjustable to acute changes in cardiac workload, for instance, during physical exercise, resulting in an increased cardiac need of substrates such as *Fa* for metabolic conversion. An increase in the value of *d*_*Alb*_, without a compensatory and counteracting change in the permeability of the endothelial cytoplasm, *P*_*ec*_, will result in an enhanced overall *Fa* permeability. Consequently, the overall *Fa* flux from capillary to cardiomyocyte increases without a change in the concentration difference of free *Fa*, the driving force of intra-cardiac *Fa* diffusion. Parameter *d*_*Alb*_ reflects a stochastic process of collision of the *AlbFa* complex with the cell membrane followed by immediate transfer of *Fa* from the binding pocket of the albumin carrier where *Fa* is bound to the outer leaflet of the phospholipid bilayer of the cell membrane, in both the microvascular compartment and the peri-vascular interstitium (Fig 1). Effective collision of the *AlbFa* complex with the cell membrane followed by instantaneous *Fa* transfer to the membrane may be enhanced by the presence of a ‘Transfer Facilitating Membrane Protein’ as hypothesized by Arts and coworkers [5]. Interaction of this putative protein with the *AlbFa* complex may, for instance, augments the dwelling time of the complex at the membrane or directs the complex into a position favorable for immediate *Fa* transfer into the membrane. Consequently, *Fa* flux from capillary to cardiomyocyte will increase while the concentration difference of unbound *Fa*, the driving force for *Fa* diffusion, remains unaltered. This consideration holds for all three albumin-containing boundary zones to be crossed: one in the capillary lumen and two in the peri-capillary interstitium. A number of membrane-associated proteins, such as *CD36*/*FAT*, *FABP*_*pm*_ and *FATP1*,*2*,*4*, as described previously [4, 25–29], may act as candidates to influence *d*_*Alb*_. Since the endothelial cell, with albumin-containing boundary zones on both sides, is the first site of intra-cardiac *Fa* transfer, the experimental identification of membrane-associated proteins in this cell type, assumed to be involved in trans-endothelial *Fa* transfer, is worth to be mentioned [26, 30, 31]. Evidence for the involvement of a 40-kD endothelial membrane-associated protein is provided by a study performed by Goresky and coworkers [11]. They showed that trans-endothelial *Fa* transfer in an isolated rat heart preparation is reduced effectively by pre-perfusion of the heart with an antibody raised against a 40-kD endothelial membrane-associated protein. Our present investigation offers a mechanistic explanation for their findings. The presence of this 40-kD protein may enhance the value of parameter *d*_*Alb*_ and, hence, the contribution of the contact pathway in delivering *Fa* to the luminal endothelial membrane.

It is of note that physical exercise associated with increased workload of the heart may enhance the concentration of the specific membrane-associated proteins mentioned above. This may result in an increased supply of *Fa* from the capillary to the cardiac muscle cells by increasing the effectiveness of the direct transfer of *Fa* from the *AlbFa* complex to cell membranes by the contact pathway, and, hence, a higher value of *d*_*Alb*_.

## Conclusions

We have presented the analysis of an extensive set of multiple indicator dilution experiments by means of a mathematical model of *Fa* transport through the coronary system and transfer from the capillaries to the cardiomyocytes handling the dynamic changes in *Fa* concentration. The experiments were performed on the intact rabbit heart *ex vivo* perfused with radiolabeled *Fa* and albumin. Our analysis clearly shows that *Fa* transfer from capillary to cardiomyocyte does not require any active, energy requiring, mechanism. Furthermore, the main resistance to intra-cardiac *Fa* transfer is located either in the extracellular boundary zones in close vicinity of cell membranes in the microvascular and interstitial compartments or in the intracellular boundary zones in the endothelial cell and cardiomyocyte or a combination of both. The relative contribution of the contact pathway. *i*.*e*., direct transfer of *Fa* from the albumin-*Fa* complex to the cell membrane, to overall *Fa* flux strongly depends on the value of the dissociation rate constant of the albumin.*Fa* complex. Our findings indicate that, in case the dissociation rate is fast, the contribution of the contact pathway is limited. However, if the dissociation rate is slow, the contribution of the contact pathway to overall intra-cardiac *Fa* flux may increase substantially. Moreover, specific membrane-associated proteins may facilitate the direct translocation of *Fa* from the *AlbFa* complex in the boundary zone to the cell membrane and, hence, increase the contribution of the contact pathway to overall intra-cardiac *Fa* transfer.

## Appendices

### Appendix 1. Completing the tail of the washout curve

To calculate the integral of the washout curve *y*(*t*), we need the complete curve. The samples of the curve cover a limited time span with the last part of the tail missing. To estimate the contribution of the tail to the integral, the time-averaged velocity profile in all coronary blood vessels is assumed to be parabolic. The tracer is considered to be injected in a short time span around time *t* = 0. Accordingly, for the tail, washout concentration *y*_*tail*_(*t*) decays proportionally with 1/*t*^2^:

$$y_{tail}(t)=\frac{C_{tail}}{t^{2}}$$ (1.1)

Symbol *C*_*tail*_ represents a constant. For the time integral of the tail with *t*>*t*_*end*_, it follows:

$$I_{tail}=\int_{t_{end}}^{\infty }y(t)dt=\frac{C_{tail}}{t_{end}}$$ (1.2)

Time *t*_*end*_ refers to the last sample. Constant *C*_*tail*_ is eliminated by combining Eq (1.1) and (1.2), rendering:

$$I_{tail}\approx y(t_{end})t_{end}$$ (1.3)

Value *y*(*t*_*end*_) is a best estimate of washout concentration at *t*_*end*_, which is derived from the last 5 sampled values. The total integral under the washout curve is found by summation of the numerically determined integral over the measuring time span and the calculated contribution *I*_*tail*_ of the tail.

### Appendix 2: Estimation of Fa extraction

In the experiments, it is assumed that *Alb* does not leave the coronary circulation. *Fa* is partially extracted with extraction fraction *E*. In the experiments, a first estimate of the extraction fraction *E*_*est*_ is derived from *Alb*(*t*) and *Fa*(*t*), representing the measured washout curves, respectively:

$$E_{est}=1-\frac{\int_{0}^{\infty }Fa(t)dt}{\int_{0}^{\infty }Alb(t)dt}$$ (2.1)

Using Eq (2.1), for some experiments, the values of *E*_*est*_ appeared negative. It is physically impossible that the true extraction fraction *E* would be negative, because the heart cannot produce radiolabeled *Fa*. Therefore, we concluded that, at least for low values of *E*, we should correct *E*_*est*_. Below, the derivation of the applied correction method is shown.

Symbol *u* represents the difference between estimated and real extraction fraction:

$$u=E_{est}-E$$ (2.2)

For likelihood *p*(*u*) we assume a Gaussian distribution around zero with standard deviation *σ*:

$$p(u)=\frac{exp(-\frac{u^{2}}{{2\sigma }^{2}})}{\sigma \sqrt{2\pi }}$$ (2.3)

When having measured *E*_*est*_, using Eq (2.2), the likelihood distribution *p*_*E*_(*Ε*) for the underlying true extraction *E* it appears:

$$p_{E}(E)=p(E_{est}-E)$$ (2.4)

Since the real extraction *E* cannot be negative, we introduced the additional condition that *p*_*E*_(*E*) = 0 for *E*<0. Thus, the most likely value *E*_*pos*_ of *E* is obtained by averaging over all allowed values of *E*:

$$E_{pos}=\frac{\int_{0}^{\infty }E\;p_{u}(E_{est}-E)dE}{\int_{0}^{\infty }p_{u}(E_{est}-E)dE}$$ (2.5)

Substituting Eq (2.3) into Eq (2.5), the solution for *E*_*pos*_ is

$$E_{pos}=E_{est}+\frac{\sigma \sqrt{2}\;exp(-\frac{{E_{est}}^{2}}{{2\sigma }^{2}})}{\sqrt{\pi }(1+erf(\frac{E_{est}}{\sigma \sqrt{2}}))}$$ (2.6)

Expression ‘erf’ indicates the error function. In Fig 8 the thus calculated *E*_*pos*_/*σ* is shown as a function of *E*_*est*_/*σ*. For *E*_*est*_ values larger than 2*σ*, *E*_*est*_ approximates *E*_*pos*_ quite accurately. For negative values of *E*_*est*_, *E*_*pos*_ is always positive.

**Fig 8:** Graphical representation of corrected extraction estimate E_pos_/σ as a function of measured extraction E_est_/σ according to Eq (2.6), where σ represents standard deviation of extraction measurement.

The value of *σ* can be estimated from the available experimental data. Considering a region around the point of zero extraction (*E* = 0), we assume that *E* is uniformly distributed for *E*>0 and equals zero for *E*<0. The distribution of *E*_*est*_ is found by convolution of the Gaussian *p*(*u*) distribution with the assumed distribution of *E*. Then, part of the values of *E*_*est*_ will be negative. The mean value of the thus found negative *E*_*est*_ values is proportional with spread *σ*. Using this property, we derived:

$$\sigma =\sqrt{\frac{8}{\pi }}\;mean({E_{est}|E}_{est}<0)$$ (2.7)

Substitution of *σ* in Eq (2.6) calculated in this way renders extraction *E*_*pos*_ as a function of the experimentally obtained values of *E*_*est*_. The correction was carried out by multiplication of the *Fa* washout curve with a factor *α*, so that Eq (2.1) will render the value *E*_*pos*_. For the correction factor, it holds:

$$\alpha =\frac{1-E_{pos}}{1-E_{est}}$$ (2.8)

### Appendix 3. Error in fit to experimental washout curve

The model simulation was fit to experimental data by minimizing the difference between the washout curves simulated by the model and determined experimentally. The objective function, representing the function that has to be minimized for best fit, was described by the sum of squared error vector components *Err*_*i*_. The latter vector was represented by the difference between sampled concentrations measured experimentally and those predicted by the mathematical model, *M*_*i*_ and *S*_*i*_, respectively, for all maximally available washout samples, *iMax*, and multiplied by a weighing function. To fit the washout peak, absolute differences were considered, implying a constant weight for all samples, as quantified by parameter *W*_*peak*_. For the tail, we considered the relative error differences more appropriate, implying the weight to be inversely proportional to washout amplitude *M*_*i*_. At the very end of the tail, noise became so prominent that the weight was reduced by introduction of noise parameter *ε*. The tail part of the washout curve has been defined as the part after the time at which 50% of the total amount of tracer was passed by. Therefore, we came to the following weight error vector:

Errj=(Sj−Mj)(Wpeakmax(Mi)+Ttail,jMj+ε)withTtail,j=max(0,−1+2∑i=1jMi∑i=1iMaxMi)andWpeak=30 (3.1)

Parameter *W*_*peak*_, representing peak weight, appeared to be not very critical. For each experiment, a large range for *W*_*peak*_ was found, causing only minor changes in the resulting fit. We have chosen *W*_*peak*_ = 30, because this value appeared to be in the range of non-critical values for all experiments. In the fitting procedure, we minimized the objective function, being the sum of squared components *Err*_*i*_.
